This article has been retracted.

# Pre-infection 25-hydroxyvitamin D3 levels and association with severity of COVID-19 illness

**DOI:** 10.1371/journal.pone.0263069

**Published:** 2022-02-03

**Authors:** Amiel A. Dror, Nicole Morozov, Amani Daoud, Yoav Namir, Orly Yakir, Yair Shachar, Mark Lifshitz, Ella Segal, Lior Fisher, Matti Mizrachi, Netanel Eisenbach, Doaa Rayan, Maayan Gruber, Amir Bashkin, Edward Kaykov, Masad Barhoum, Michael Edelstein, Eyal Sela

**Affiliations:** 1 Department of Otolaryngology, Head and Neck Surgery, Galilee Medical Center, Nahariya, Israel; 2 Azrieli Faculty of Medicine, Bar-Ilan University, Safed, Israel; 3 Sackler Faculty of Medicine, Tel Aviv University, Tel Aviv, Israel; 4 Statistical Analysis Division, Galilee Medical Center, Nahariya, Israel; 5 Computer Data Division, Galilee Medical Center, Nahariya, Israel; 6 Endocrinology Unit, Galilee Medical Center, Nahariya, Israel; 7 Geriatric Medicine Department, Galilee Medical Center, Nahariya, Israel; 8 Galilee Medical Center, Nahariya, Israel; University of Hong Kong, HONG KONG

## Abstract

**Objective:**

Studies have demonstrated a potential correlation between low vitamin D status and both an increased risk of infection with SARS-CoV-2 and poorer clinical outcomes. This retrospective study examines if, and to what degree, a relationship exists between pre-infection serum 25-hydroxyvitamin D (25(OH)D) level and disease severity and mortality due to SARS-CoV-2.

**Participants:**

The records of individuals admitted between April 7^th^, 2020 and February 4^th^, 2021 to the Galilee Medical Center (GMC) in Nahariya, Israel, with positive polymerase chain reaction (PCR) tests for SARS-CoV-2 (COVID-19) were searched for historical 25(OH)D levels measured 14 to 730 days prior to the positive PCR test.

**Design:**

Patients admitted to GMC with COVID-19 were categorized according to disease severity and level of 25(OH)D. An association between pre-infection 25(OH)D levels, divided between four categories (deficient, insufficient, adequate, and high-normal), and COVID-19 severity was ascertained utilizing a multivariable regression analysis. To isolate the possible influence of the sinusoidal pattern of seasonal 25(OH)D changes throughout the year, a cosinor model was used.

**Results:**

Of 1176 patients admitted, 253 had records of a 25(OH)D level prior to COVID-19 infection. A lower vitamin D status was more common in patients with the severe or critical disease (<20 ng/mL [87.4%]) than in individuals with mild or moderate disease (<20 ng/mL [34.3%] *p* < 0.001). Patients with vitamin D deficiency (<20 ng/mL) were 14 times more likely to have severe or critical disease than patients with 25(OH)D ≥40 ng/mL (odds ratio [OR], 14; 95% confidence interval [CI], 4 to 51; *p* < 0.001).

**Conclusions:**

Among hospitalized COVID-19 patients, pre-infection deficiency of vitamin D was associated with increased disease severity and mortality.

## Introduction

Vitamin D is most often recognized for its role in bone health, but a low vitamin D status has been associated with a range of autoimmune, cardiovascular, and infectious diseases due to its role as an essential immunologic mediator [1]. Experimental laboratory evidence evaluating the impact of vitamin D on immunological responses has shown inhibitory effects on the production of pro-inflammatory cytokines, including TNF-alpha and IL-6, by various mechanisms, including down-regulating viral-induced NFkB activation [2].

Vitamin D deficiency is a global health problem, and its high prevalence in the Middle East has been established [3]. Epidemiological risk factors for vitamin D deficiency include greater skin pigmentation, low sun exposure, use of skin-covering clothes, and a diet low in fish and dairy products. Studies have previously demonstrated that social habits in specific ethnic groups and a preference to wear long clothing outdoors are independent risk factors for vitamin D deficiency, particularly among women [4]. Consistent with laboratory data, clinical studies have established an association between low 25-hydroxyvitamin D (25(OH)D) levels and an increased risk of acquiring influenza and respiratory viruses [5]. Meta-analyses of randomized controlled trials conducted between 2007 and 2020 suggest that vitamin D supplementation reduced the risk of acute respiratory infection as compared with placebos [6].

COVID-19 is an acute respiratory infection caused by the SARS-CoV-2 virus, theorized to have emerged in China in December 2019, which rapidly developed into a global pandemic. Factors associated with poorer COVID-19 prognoses include geographic location in northern countries, older age, darker skin pigmentation, BAME ethnicity (Black and minority ethnic groups), male sex, obesity, and history of preexisting conditions such as diabetes and hypertension; these risk factors are also independently associated with vitamin D deficiency [7].

As with other respiratory infections, a link between vitamin D deficiency and COVID-19 infection is emerging [8, 9]. Low serum 25(OH)D levels among hospitalized COVID-19 patients have also been linked with increased disease severity and poorer clinical outcomes [10]. In addition, hospitalized COVID-19 patients have been shown to present lower mean and median levels of 25(OH)D than the general population and COVID-19 outpatients [11]. However, serum 25(OH)D is often measured during hospitalization for COVID-19. When this is the case, determining the direction and temporality of the association between acute COVID-19 disease and low 25(OH)D serum levels is a challenge. In other words, it is difficult to ascertain a definitive causative effect of baseline vitamin D status on a clinical presentation during active COVID-19 infection.

To better understand the temporal sequence between low 25(OH)D levels and their association with the severity of acute COVID-19 disease, we determined whether the severity of disease among patients admitted with acute COVID-19 correlated with their most recent pre-infection 25(OH)D serum levels. By utilizing the pre-infection 25(OH)D values, meaning those obtained from the patient’s medical records, and applying a novel cosinor model technique to predict annual and monthly 25(OH)D levels, we demonstrate statistically significant and consistent findings of an association between lower 25(OH)D levels and higher COVID-19 disease severity.

## Methods

### 1. Participants

This was a retrospective study. Prior to study initiation, ethical approval was granted by the Research Ethics Committee of the Galilee Medical Center 0204-20-NHR. Data collection included existing non-identifiable patient medical records, and informed consent was exempted for this study. Inclusion criteria were adult patients with PCR-confirmed COVID-19 infection admitted to Galilee Medical Center (GMC) between April 7^th^, 2020, and February 4^th^, 2021. Patients under the age of 18 years old were excluded from this study.

### 2. Patient and public involvement

Patients and the public were not involved in the design or conduct of this study and did not contribute to the analysis of results.

### 3. Measurement

COVID-19 infection was confirmed by two independent positive polymerase chain reaction (PCR) tests. Clinical data collected during the inpatient hospital stay at Galilee Medical Center included length of hospitalization in days, the severity of illness (mild, moderate, severe, and critical, as determined by the WHO definition of COVID-19 disease severity (WHO/2019-nCoV/clinical/2020.5)), mortality during hospitalization, and comorbidities (COPD, chronic heart failure, chronic ischemic heart disease, chronic renal disease, diabetes, and hypertension). Additional demographic characteristics included age, ethnicity, and BMI (S1 Dataset).

Disease severity was calculated at the point of highest severity during the patient’s inpatient stay; as an example, a patient who arrived at the hospital in mild condition but decompensated to a critical condition during admission would be classified as having had a critical illness. Each patient’s 25(OH)D level was collected from their respective electronic medical records 14 to 730 days prior to COVID-19 diagnosis. The most recent 25(OH)D level from prior to infection with COVID-19 was collected via a standardized commercial 25(OH)D kit assay. Patients with previous 25(OH)D measurements had likely been tested either as part of a routine blood workup or following a clinical suspicion for vitamin D deficiency. We did not have access to data regarding whether patients had been treated for vitamin D deficiency. Patients’ 25(OH)D levels were divided into four universally accepted categories: deficient (below 50 nmol/L or 20 ng/mL), insufficient (50 nmol/L to 75 nmol/L or 20–29.9 ng/mL), adequate (75–99.75 nmol/L or 30–39.9 ng/mL), and high-normal (equal to or above 187.5 nmol/L or 40 ng/mL).

### 4. Analysis

Continuous variables were presented as the mean ± standard deviation or as median and range values. Qualitative variables were presented as frequencies and percentages.

A univariate analysis provided comparisons of continuous variables among groups examined with either the ANOVA, Kruskal-Wallis test, Independent sample t-test, or Mann-Whitney test. Those tests were chosen according to the number of the compared groups, the sample size of the groups, and the variables’ distribution shape. Ordinal variables were compared among the groups with the Kruskal-Wallis test or the Mann-Whitney test, chosen according to the number of the compared groups, and categorical variables using the Pearson’s chi-square test or the Fisher’s exact test (if expectancy < 5). The intensity of the correlation between BMI and 25(OH)D (which are both categorical variables) was examined with Crammer’sV. Correlations between 25(OH)D level and COVID-19 disease severity (which are continuous variable and variable measured on the ordinal scale, respectively) were examined with the Spearman’s correlation coefficient test.

For the multivariable analysis, a multivariable logistical regression model (with the backward elimination method) was performed in order to examine the correlation between the 25(OH)D level and COVID-19 disease severity as the dependent variable. Combined severity categories were used (‘mild/moderate’ and ‘severe/critical’) consistent with the required specification of this model to include dichotomous dependent variable. This model was adjusted to several variables such as age, gender, BMI, and comorbidities. Those variables have been included in the multivariable model as independent variables because they were found to be significant in the univariate analysis or due to theoretical clinical considerations. Hosmer and Lemshow’s goodness of fit test was utilized, and the odds ratio (OR) and 95% confidence intervals (CI) were presented.

We took into special consideration the seasonal variations in circulating 25(OH)D concentrations. Several reports have established that 25(OH)D follows a sinusoidal pattern, leading to misclassifications of 25(OH)D if seasonality is not accounted for in statistical analyses [12–18]. To eliminate the occurrence of seasonal variability, we approximated seasonal differences by using a cosinor model to predict both annual and monthly mean 25(OH)D concentrations for patient’s single 25(OH)D measurement taken within the 14–730 days prior to positive COVID-19 results. The cosinor model is a validated tool to predict the mean annual and monthly 25(OH)D concentrations from a single measurement [14–20].

### 5. The cosinor model

Consistent with previously published research which determined that 25(OH)D values follow an annual sinusoidal pattern, our study population’s median and mean 25(OH)D concentrations were lowest in January and February (late Winter) and were highest in July and August (mid-late Summer). Therefore, we examined whether a cosinor model is an adequate tool to evaluate our data. Time was presented in months.

In general, the cosinor model transforms the time variable (the month) into sine and cosine terms and then fits a linear regression model in which the dependent variable is the pre-infection 25(OH)D concentration, and the sine and cosine terms are the independent variables. These two terms represent the sinusoidal pattern of the curve [16–18].

The cosinor model hypothesis of an amplitude equal to zero was rejected [F (2, 250) = 3.10, *p* = 0.047], MSE = 9.87, and the mean bias (the observation minus the predicted values) is 0.53. The required assumptions of the cosinor model (particularly the equal variance assumption, the residuals normality assumption, and the independence of residuals) were examined with a scatter plot (residuals versus the predicted values), a histogram for the residuals, Q-Q plot, Kolmogrov-Smirnov test for normality, and the Run test. We did not find significant violations of the model’s assumptions requiring a rejection of the cosinor model.

Along with the cosinor model, 25-hydroxyvitamin D (25(OH)D) levels follow a sine wave over time, characterized by the mesor (the mean level of oscillation), phase (the location of the peaks along the time axis), acrophase (referring to the angle of the phase) and an amplitude (an estimate of seasonal variation, defined as the distance from the mean to the highest or lowest value of the sine curve (the peak-trough on the y-axis) divided by two. Note that the mesor, the amplitude, and the phase can be achieved or calculated from the regression coefficients directly [16–18].

### 6. The model’s prediction

To predict the mean annual 25(OH)D concentration for each specific patient, we used the model’s output, the predictive value of the cosinor model. A manual method of calculating this predicted value is to add to the mean 25(OH)D value for the entire sample (the mesor) the difference between the observed 25(OH)D pre-infection measurement for a specific patient and the monthly 25(OH)D mean level, at the month in which the measurement was collected, calculated according to the sine curve with Eq 2, below.

As an example, an individual may have a 25(OH)D concentration of 40 ng/mL in January and a sine curve in January containing a mean value of 30 ng/mL. With a cosinor model estimating the annual mean of the whole study population (mesor) as 20 ng/mL, the resulting equation would be: 20 ng/mL + (40 ng/mL– 30 ng/mL) = 30 ng/mL, which is an estimate of this individual’s annual mean 25(OH)D level [17].

The equation to predict the annual mean 25(OH)D for each patient (Eq 1) is written as follows:

**Eq 1** [17]: Predicted 25(OH)D annual mean (patient-specific)

$$pVitD_{\mathrm{annual}}=M+(p{\mathrm{VitD}}_{\mathrm{preinfection}}-m{\mathrm{VitD}}_{\mathrm{preinfection}})$$

Eq 1 abbreviations:

pVitD_*annual*_ = Predicted 25(OH)D annual mean (patient-specific)

M = Mesor

pVitD_*preinfection*_ = Pre-infection patient’s 25(OH)D measurement (patient-specific)

mVitD_*preinfection*_ = Predicted 25(OH)D monthly mean at the measurement date, using Eq 2 (month-specific)

The equation to predict mean 25(OH)D level for each month (Eq 2) is written as follows:

**Eq 2:** Predicted 25(OH)D monthly mean (month-specific)

$$m\mathrm{Vit}D=M+A\times (\mathrm{Cos}(\frac{2\times \pi \times m}{\mathrm{Period}}+\mathrm{Phi}))$$

Eq 2 abbreviations:

mVitD = Prediction of 25(OH)D mean per month

M = Mesor

A = Amplitude

m = Month

Period = 12

Phi = Acrophase

The calculated cosinor model of 25(OH)D values, following a sine wave, had a mean of 26.33 ng/mL (mesor) (SD = 1.26) with an estimated peak-trough difference (amplitude) in 25(OH)D concentration of 4.55 ng/mL (SD = 1.84) and an acrophase of –3.25 (SD = 0.39) (Fig 1).

**Fig 1:** The cosinor 25(OH)D model for all months. The predicted 25(OH)D mean value of each month through the annum can be extracted from the graph. This figure demonstrates the predicted peak of 25(OH)D concentration in June and the expected trough in December. The predicted 25(OH)D mean value of each month can be utilized to predict the 25(OH)D for the hospitalization month of any given patient (Eq 3). M = mesor, A = amplitude, P = Phase.

An accurate prediction of 25(OH)D level at a specific date (e.g. as at the hospitalized date) for each patient can be achieved if more than one 25(OH)D measurement exists for each patient or if a multivariable model is adopted; the additional independent variables, except the month, must be variables which can influence the amplitude or the phase.

If lacking in multiple measurements, the alternative method is to predict each patient’s 25(OH)D level during the hospitalized month with the methodology we employed, written as follows:

With the cosinor model, we can obtain a prediction of the seasonal variation of the sample and then assume that this variation throughout the year is identical for all the participants in the sample. If, for example, the cosinor model predicted that the 25(OH)D monthly mean concentration was 60 ng/mL in June and 40 ng/mL in January, the difference is 20 ng/mL. Therefore, in an individual with a 25(OH)D measurement of 75 ng/mL in June, if we wish to predict this individual’s January 25(OH)D level we subtract 20 ng/mL with the resulting level of 55 ng/mL. The equation to predict 25(OH)D concentration for each specific patient at the hospitalization date (Eq 3) is written as follows:

**Eq 3:** Predicted 25(OH)D for the hospitalization month (patient-specific)

$$p\mathrm{Vit}D_{\mathrm{hospitalization}}=p\mathrm{Vit}D_{\mathrm{preinfection}}-(m\mathrm{Vit}D_{\mathrm{preinfection}}-m\mathrm{Vit}D_{\mathrm{hospitalization}})$$

Eq 3 abbreviations:

pVitD_*hospitalization*_ = Prediction of 25(OH)D for the month of hospitalization (patient-specific)

pVitD_*preinfection*_ = Pre-infection patient’s 25(OH)D measurement (patient-specific)

mVitD_*preinfection*_ = Predicted 25(OH)D monthly mean at the measurement date, using Eq 2 (month-specific)

mVitD_*hospitalization*_ = Predicted 25(OH)D monthly mean for the month of hospitalization, using Eq 2 (month-specific).

We present, altogether, the pre-infection 25(OH)D values from each patient’s date of collection as well as the prediction of the cosinor model for the annual mean and for the month in which the patient was hospitalized.

We used a statistical significance threshold of P<0.05, and a two-sided p-value was presented unless otherwise stated. The analysis was performed using the IBM SPSS Statistic software, version 27.0. For the cosinor model adaption, we used the R software version 1.4.1717 with packages including the cosinor, cosinor2, card, and psych packages.

## Results

Of 1176 individuals admitted for COVID-19 at the Galilee Medical Center between April 7^th^, 2020, and February 4^th^, 2021, 253 (21.5%) individuals (mean age 63.3 [SD = 18.6] years; 144 [56.9%] women) had historical 25(OH)D levels obtained between 14 and 730 days before their first positive COVID-19 test (Table 1).

**Table 1:** Characteristics of hospitalized COVID-19 patients stratified by pre-infection 25(OH)D level measured 14 to 730 days before positive COVID-19 test.

		No. (%)					
Characteristics		Most recent 25(OH)D level (ng/mL) before COVID-19 test (N = 253)				*p* value 2-sided (between groups)	*p* value 2-sided (<20 compared with ≥20)
		<20	20–29.9	30–39.9	≥40		
No. of patients		133	36	44	40		
Age, y							
	mean (std)	68.4 (15.9)	62.2 (17.9)	55.7 (20.7)	57.8 (21.0)	*p* < 0.001§	*p* < 0.001^
	Range	27.3–95.8	22.7–92.7	19.3–92.7	19.8–90		
	<50	18 (13.5)	8 (22.2)	18 (40.9)	17 (42.5)	*p* < 0.001§	*p* < 0.001†
	50–64	36 (27.1)	14 (38.9)	10 (22.7)	6 (15.0)		
	≥65	79 (59.4)	14 (38.9)	16 (36.4)	17 (42.5)		
Sex							
	Female	69 (51.9)	18 (50.0)	30 (68.2)	27 (67.5)	*p* = 0.10	*p* = 0.10
	Male	64 (48.1)	18 (50.0)	14 (31.8)	13 (32.5)		
Ethnicity							
	Arabs	83 (64.3)	16 (44.4)	33 (76.7)	19 (47.5)	*p* = 0.006	*p* = 0.30
	Non-Arabs	46 (35.7)	20 (55.6)	10 (23.3)	21 (52.5)		
COVID-19 disease severity category (WHO)							
	Mild	7 (5.3)	8 (22.2)	37 (84.1)	28 (70.0)	*p* < 0.001 §	*p* < 0.001 †
	Moderate	50 (37.6)	24 (66.7)	3 (6.8)	9 (22.5)		
	Severe	64 (48.1)	3 (8.3)	4 (9.1)	3 (7.5)		
	Critical	12 (9.0)	1 (2.8)	0 (0.0)	0 (0.0)		
BMI							
	mean (std)						
	<30	98 (73.7)	32 (88.9)	34 (77.3)	34 (85.0)	*p* = 0.163	*p* = 0.07
	≥30	35 (26.3)	4 (11.1)	10 (22.7)	6 (15.0)		
Mortality during hospitalization							
	Yes	34 (25.6)	1 (2.8)	1 (2.3)	2 (5.0)	*p* < 0.001	*p* < 0.001
	No	99 (74.4)	35 (97.2)	43 (97.7)	38 (95.0)		
Comorbidities							
	COPD	82 (61.7)	15 (41.7)	20 (45.5)	18 (45.0)	*p* = 0.048	*p* = 0.006
	Chronic heart failure	16 (12.0)	3 (8.3)	1 (2.3)	2 (5.0)	*p* = 0.211‡	*p =* 0.07
	Chronic ischemic heart disease	16 (12.0)	3 (8.3)	3 (6.8)	1 (2.5)	*p* = 0.316‡	*p* = 0.124
	Chronic renal disease	17 (12.8)	5 (13.9)	3 (6.8)	3 (7.5)	*p* = 0.60‡	*p* = 0.425
	Diabetes	56 (42.1)	9 (25.0)	12 (27.3)	13 (32.5)	*p* = 0.125	*p* = 0.03
	Hypertension	82 (61.7)	16 (44.4)	21 (47.7)	18 (45.0)	*p* = 0.092	*p* = 0.02

Abbreviations: BMI, body mass index (calculated as weight in kilograms divided by height in meters squared); COVID-19, coronavirus disease 2019; Patient data includes COVID-19 admission between Apr 7^th^, 2020 to Feb 4^th^, 2021 who had serum 25(OH)D level measured between 14 to 730 days before positive PCR test. Most recent 25(OH)D level was depicted for the purpose of the study.

*p* values were determined using the Pearson Chi-Square test unless mentioned otherwise.

^ *p* values were determined using the independent t-test.

‡ *p* values were determined using the Fisher-Freeman-Halton Exact Test.

§ *p* values were determined using Kruskal-Wallis Test.

† *p* values were determined using Mann-Whitney Test.

Data were analyzed both directly and through the cosinor model; the “direct” method included the pre-infection 25(OH)D levels (i.e., if a patient’s 25(OH)D level was 50 ng/mL on the date of examination, this was the measurement used).

Tables 1 and 2 include the direct method while the cosinor model-predicted annual and monthly 25(OH)D values at the hospitalization dates are presented in Table 3.

**Table 2:** Characteristics of hospitalized COVID-19 patients and their pre-infection measurement of 25(OH)D levels, stratified by COVID-19 disease severity category.

		No. (%)				*p* value 2-sided (between groups)	*p* value 2-sided (severe/critical vs. mild/moderate disease)
Characteristics		COVID-19 disease severity category (WHO)					
		Mild	Moderate	Severe	Critical		
No. of patients		80 (31.6)	86 (34.0)	74 (29.2)	13 (5.1)		
Age, y							
	mean (std)	53.1 (19.8)	64.2 (16.4)	72.1 (14.7)	76.0 (11.6)	*p* < 0.001§	*p* < 0.001^
	Range	19.3–90.0	30.4–95.9	28.8–94.9	52.6–92.1		
	<50	36 (45.0)	19 (22.1)	6 (8.1)	0 (0.0)	*p* < 0.001§	*p* < 0.001†
	50–64	20 (25.0)	27 (31.4)	18 (24.3)	1 (7.7)		
	≥65	24 (30.0)	40 (46.5)	50 (67.6)	12 (92.3)		
Sex							
	Female	51 (63.7)	53 (61.6)	35 (47.3)	5 (38.5)	*p* = 0.08	*p* = 0.01
	Male	29 (36.3)	33 (38.4)	39 (52.7)	8 (61.5)		
Ethnicity							
	Arabs	49 (62)	55 (64.0)	37 (52.9)	10 (76.9)	*p* = 0.30	*p* = 0.34
	Non-Arabs	30 (38)	31 (36)	33 (47.1)	3 (23.1)		
Pre-infection 25(OH)D level (ng/mL) evaluated 14–730 days before positive COVID-19 test							
	median	34.2	18.9	11.3	10.0		
	Range	10.0–83.6	5.6–158	5.7–67.4	6.2–22.2		
	<20	7 (8.8)	50 (58.1)	64 (86.5)	12 (92.3)	*p* < 0.001 §	*p* < 0.001†
	20–29.9	8 (10)	24 (27.9)	3 (4.1)	1 (7.7)		
	30–39.9	37 (46.2)	3 (3.5)	4 (5.4)	0 (0.0)		
	≥40	28 (35.0)	9 (10.5)	3 (4.0)	0 (0.0)		
BMI							
	mean (std)	27.5 (5.9)	27.6 (4.5)	29.2 (5.1)	32(4.3)		
	<30	66 (82.5)	69 (80.2)	55 (74.3)	8 (61.5)	*p* = 0.28‡	*p* = 0.11
	≥30	14 (17.5)	17 (19.8)	19 (25.7)	5 (38.5)		
Mortality during hospitalization		0 (0.0)	1 (1.2)	26 (35.1)	11 (84.6)	*p* < 0.001‡	*p* < 0.001

Abbreviations: BMI, body mass index (calculated as weight in kilograms divided by height in meters squared); COVID-19. Patients included were those admitted for COVID-19 between Apr 7^th^, 2020 and Feb 4^th^, 2021 who had serum 25(OH)D level measured between 14–730 days before the positive COVID-19 test. The most recent 25(OH)D result was used for the purpose of the study.

P values were determined using the Pearson Chi-Square test unless mentioned otherwise.

^ *p* values were determined using the independent t-test.

‡ P values were determined using the Fisher-Freeman-Halton Exact Test.

§ P values were determined using Kruskal-Wallis Test.

† P values were determined using Mann-Whitney Test.

**Table 3:** 25(OH)D level stratified by COVID-19 disease severity category before and after cosinor correction models for the annual mean as well as each patient’s date of hospitalization.

		No. (%)				*p* value 2-sided (between groups)	*p* value 2-sided (severe/critical vs. mild/moderate disease)
Characteristics		COVID-19 disease severity category (WHO)					
		Mild	Moderate	Severe	Critical		
Pre-infection 25(OH)D level (ng/mL) evaluated 14–730 days before positive COVID-19 test							
	median	34.2	18.9	11.3	10.0		
	<20	7 (8.8)	50 (58.1)	64 (86.5)	12 (92.3)	*p* < 0.001 §	*p* < 0.001†
	20–29.9	8 (10)	24 (27.9)	3 (4.1)	1 (7.7)		
	30–39.9	37 (46.2)	3 (3.5)	4 (5.4)	0 (0.0)		
	≥40	28 (35.0)	9 (10.5)	3 (4.0)	0 (0.0)		
Predicted 25(OH)D level (ng/mL) annual mean correction based on the cosinor model [Eq 1]							
	median	36.2	18.1	11.1	10.9		
	<20	7 (8.8)	46 (53.5)	64 (86.5)	11 (84.6)	*p* < 0.001 §	*p* < 0.001 †
	20–29.9	11 (13.8)	26 (30.2)	3 (4.1)	2 (15.4)		
	30–39.9	35 (43.8)	5 (5.8)	4 (5.4)	0 (0.0)		
	≥40	27 (33.8)	9 (10.5)	3 (4.1)	0 (0.0)		
Predicted 25(OH)D level (ng/mL) corrected to the hospitalization date based on the cosinor model [Eq 3]							
	median	36.1	19.4	13.0	11.8		
	<20	6 (7.5)	52 (60.5)	63 (85.1)	11 (84.6)	*p* < 0.001 §	*p* < 0.001 †
	20–29.9	12 (15)	18 (20.9)	4 (5.4)	2 (15.4		
	30–39.9	33 (41.3)	8 (9.3)	4 (5.4)	0 (0.0)		
	≥40	29 (36.3)	8 (9.3)	3 (4.1)	0 (0.0)		

§ P values were determined using Kruskal-Wallis Test.

† P values were determined using Mann-Whitney Test.

In the direct methodology, of the 253 individuals with pre-infection 25(OH)D levels, 133 (52.5%) had a level less than 20 ng/mL, 36 (14.2%) had 20 to less than 30 ng/mL, 44 (17.3%) had 30 to less than 40 ng/mL, and 40 (15.8%) had 40 ng/mL or greater (Table 1). Mortality among patients with sufficient vitamin D levels was 2.3%, in contrast to the vitamin D deficient group’s 25.6% mortality rate (*p* <0.001) (Table 1). Stratified by COVID-19 disease severity, a lower 25(OH)D status was more common in patients with severe or critical disease (<20 ng/mL: 76 of 87 individuals [87.4%]) than individuals with mild or moderate disease (<20 ng/mL: 57 of 166 individuals [34.3%] *p* < 0.001) (Table 2).

Following the cosinor model, we predicted the patients’ vitamin D status either for annual mean values or toward the month of hospitalization. With reclassified categorizations of vitamin D level stratifications, results between the direct and cosinor models were consistently similar, and the deviations were between neighboring categories. The accuracy between the pre- and post-cosinor model predictive values was 85% for mean 25(OH)D annual correction and 83% for the patient’s hospitalization month correction. Moreover, the proportion of patients with vitamin D deficiency before cosinor correction was 53% as compared to 51% and 52% following 25(OH)D correction for annual mean or for the hospitalization month, respectively.

According to the multivariable analysis, 25(OH)D was found to be correlated with COVID-19 illness severity with respect to both the pre-infection values as well as the cosinor-predicted values (Table 4).

**Table 4:** Multivariable logistic regression analysis of possible predictors of severe or critical COVID-19 disease among hospitalized patients with a pre-infection measurement of 25(OH)D level. The multivariable analyses before and after cosinor correction models for the annual mean as well as each patient’s date of hospitalization are shown. This is the final step in the logistic regression (backward elimination).

					Pre-infection 25(OH)D level (ng/mL)			Predicted 25(OH)D (ng/mL) annual mean			Predicted 25(OH)D level (ng/mL) corrected to the hospitalization date		
					Values obtained from patient’s chart			Values corrected according to cosinor model (Eq 1)			Values corrected according to cosinor model (Eq 3)		
	Mild/moderate cases		Severe/critical cases		OR	95%CI	*p* value	OR	95%CI	*p* value	OR	95%CI	*p* value
variable	N	%	N	%									
25(OH)D levels							*p* < 0.001			*p* < 0.001			*p* < 0.001
≥40	37	92.5%	3	7.5%	baseline			baseline			baseline		
30–39.9	40	90.9%	4	9.1%	1.45	0.29–7.25	*p* = 0.65	1.23	0.25–6.20	*p* = 0.80	1.11	0.22–5.48	*p* = 0.90
20–29.9	32	88.9%	4	11.1%	1.32	0.26–6.78	*p* = 0.74	1.36	0.29–6.42	*p* = 0.70	2.48	0.55–11.26	*p* = 0.24
<20	57	42.9%	76	57.1%	14	4–51	*p* < 0.001	14.49	4.01–51.73	*p* < 0.001	12.43	3.52–43.85	*p* < 0.001
Mean age, years (std)	58.9 (18.9)		72.7 (14.3)		1.04	1.02–1.06	*p* = 0.001	1.04	1.02–1.06	*p* < 0.001	1.03	1.007–1.05	*p* = 0.01
Diabetic													
yes	45	50%	45	50%	2.03	1.04–3.97	*p* = 0.04	2.00	1.02–3.90	*p* = 0.04	(/)		
no	121	74.2%	42	25.8%	baseline			baseline					
COPD					(/)			(/)					
yes	71	52.6%	64	47.4%							2.01	0.97–4.14	*p* = 0.06
no	95	80.5%	23	19.5%							baseline		
Constant					0.004		*p* < 0.001	0.005		*p* < 0.001	0.009		*p* < 0.001

Multivariable logistic regression analysis, backward elimination method. Dependent variable: COVID-19 disease severity (severe or critical vs. mild or moderate). The variables included in step 1 of this model were age, sex (male), BMI, and presence of chronic obstructive pulmonary disease (COPD), chronic heart failure (CHF), chronic ischemic heart disease (CIHD), chronic renal failure (CRF), or diabetes. Included are the 25(OH)D levels [Pre-infection 25(OH)D level obtained from patient’s chart; predicted 25(OH)D annual mean corrected according to cosinor model (Eq 1); and predicted 25(OH)D level (ng/mL) corrected to the hospitalization date corrected according to cosinor model (Eq 3)]. OR = odds ratio; CI = confidence interval; (/) Removed in the last step of backward elimination.

The variables included in step 1 of this multivariable regression model (not presented) were age, sex (male), BMI, and comorbidities. The final model represents the last step of the backward elimination process following the adjustment of confounding factors (Table 4).

Based on the pre-infection values, patients with vitamin D deficiency (<20 ng/mL) were 14 times more likely to have severe or critical disease than patients with 25(OH)D ≥40 ng/mL (OR, 14; 95% CI, 4 to 51; *p* < 0.001) (Table 4). An independent risk factor for severe COVID-19 disease was age (Table 4). While VitD and age were consistently found as risk factors for increased COVID-19 disease severity, one multivariate analysis found pre-existing COPD associated with COVID-19 disease severity while another multivariate analysis found diabetes as an association.

A comparison of pre-infection 25(OH)D values among COVID-19 disease severity categories demonstrated a progressive decrease in levels of 25(OH)D as the disease severity increased (Fig 2). A significant difference in 25(OH)D level was found between mild compared with moderate disease categories (*p* = 0 .001) and moderate compared with severe (*p* = 0.002) (in the mild group, 8.8% had a level less than 20 ng/mL, as well as 58.1% in the moderate group, and 86.5% in the severe patients) (Fig 2 and Table 1). No difference between severe and critical individuals with regards to 25(OH)D (*p* = 0.41) was observed (Fig 2).

**Fig 2:** Box-and-whisker plots of the most recent pre-infection serum 25(OH)D levels before hospitalization were collected as a baseline (N = 253). The mean vitamin level was compared between the four categories of COVID-19 disease severity as determined by the WHO definition (WHO/2019-nCoV/clinical/2020.5). A Kruskal-Wallis test for multiple-category comparison shows a significant difference between groups *p* < 0.001. A Mann-Whitney test compared vitamin D mean rank of two neighboring categories sequentially; mild compared with moderate (mean difference, 12.96 ng/mL; [Rank difference 26.65] *p* < 0.001); moderate compared with severe (mean difference, 10.72 ng/mL [Rank difference 23.08]; *p* < 0.002); Severe compared with Critical (mean difference, 3.96 ng/mL [Rank difference 6.33]; *p* = 0.40). The boxes present the range of vitamin D values within the interquartile range (50% of the cases). The whiskers outside the box mark the most upper and lower values within 1.5 times the interquartile range. Outliers’ values in each group are represented with empty circles.

While both age and pre-infection vitamin D baseline status are independent predictors of increased disease severity, further analysis found a significant correlation between vitamin D deficiency when stratifying patients into three age groups (<50, 50–64, ≥65) (Fig 3). The strongest correlation between lower 25(OH)D levels and COVID-19 disease severity was seen in ≥50 years old patients (r = – 0.74; *p* < 0.001 for ages 50–64 years; r = – 0.72; *p* < 0.001 for ages ≥65). In patients under 50 years of age, COVID-19 severity was still correlated with vitamin D deficiency but to a lesser extent (r = – 0.66; *p* < 0.001). Similar trends were found with the cosinor model correction (with the mean annual and with the correction for the month that a person was hospitalized).

**Fig 3:** Correlation between pre-infection vitamin D deficiency status and COVID-19 disease severity stratified by three different groups of age (<50, 50–64, ≥65). The severity of illness (critical, severe, moderate, and mild, as determined by the WHO definition of COVID-19 disease severity (WHO/2019-nCoV/clinical/2020.5)). The regression fit for each age group is shown. Values that are more than two SD away from the regression fit to the rest of the data were omitted from the analysis (applicable for two values appear on <50 yr graph that omitted from regression fit calculation).

Finally, among patients with a BMI <30, 49.5% have a 25(OH)D <20 ng/mL compared to 63.6% among patients with a BMI ≥ 30+ (*p* = 0.07, 2-sided; *p* = 0.04, 1-sided). The intensity of the correlation between BMI and vitamin D deficiency does not indicate a strong correlation (Crammer’V = 0.117). As a result, 25(OH)D was not, and cannot be, used as a surrogate value for BMI.

## Discussion

In this retrospective single-institution study, we demonstrate a correlation between insufficient 25-hydroxyvitamin D (25(OH)D) level prior to COVID-19 infection and increased COVID-19 disease severity and mortality during hospitalization.

The vital role of vitamin D during the COVID-19 pandemic has been highlighted beyond its well-known benefit for bone and muscle health as a regulatory component of the innate and adaptive immune responses during viral infections [21]. Other hallmarks of COVID-19 disease have been linked with vitamin D status, including the cytokine storm that portends acute respiratory distress syndrome [22, 23]. Several studies demonstrated the association of vitamin D deficiency in a patient’s history with an increased risk for positive COVID-19 test results [9]. Existing research has suggested a correlation between low 25(OH)D levels upon admission as a predictor of poorer COVID-19 disease outcomes [11]. However, a low level of serum 25(OH)D measured during the acute COVID-19 infection may reflect a consequence of chronic inflammation rather than an underlying cause [24].

To overcome this possible bias, we followed a previously described methodology of using the most recent historical vitamin D prior to COVID-19 illness [25]. With this approach, the vitamin D values obtained assuredly preceded COVID-19 infection and reflect the potential effect of vitamin D serum status on COVID-19 disease severity and mortality. To further ensure a high degree of accuracy with regards to 25(OH)D levels preceding the infection date, we performed our analyses using the pre-infection value as well as predicted values from a cosinor model, which considers the cycles of serum vitamin D values across the seasons of the year. The methodologies of use for this cosinor model, based on the sinusoidal pattern of 25(OH)D values throughout the annum, is described in detail within our Methods section. With the sine curve, we predicted the 25(OH)D level at patient admission date according to the previous measurements taken at any pre-admission time point. For the purposes of our study, the relevant unit of time was a month.

For both the pre-infection and cosinor-predicted values for each hospitalization date, we found that lower 25(OH)D levels were associated with greater disease severity and mortality. While 48.1% of vitamin D deficient (<20 ng/mL) patients (pre-infection 25(OH)D level) had severe disease courses, less than 10% of patients with vitamin D levels ≥20 ng/mL had severe courses. While the mortality of patients who had 25(OH)D vitamin D levels ≥20 ng/mL was 5% or lower, the mortality of vitamin D deficient patients (<20 ng/mL) was much higher, at 25.6%.

Older age is associated with both vitamin D deficiency and poorer COVID-19 outcomes. We performed a multivariable analysis which adjusted for age as a confounder, demonstrating that pre-infection vitamin D deficiency increased the risk of severe COVID-19 disease, at any group of age. Reduced 25(OH)D levels in younger COVID-19 inpatients may suggest an increased hospitalization risk due to COVID-19 illness in this group with severely low 25(OH)D while older patients remain at increased risk of hospitalization for COVID-19, even with higher levels of the vitamin D deficiency range.

The high percentage of vitamin D deficiency among Israeli Arabs (64.3% of patients with vitamin D <20 ng/mL) compared with Israeli non-Arabs (35.7% of patients with vitamin D <20 ng/mL) was consistent with previous research demonstrating high rates of vitamin D deficiency in Arabs, including in Arab American and Arab-European populations [26, 27]. Mechanisms for vitamin D insufficiency among different ethnic groups are subject to investigation and span across inherited and environmental factors or a combination of both [28, 29]. A recent study among United Arab Emirates (UAE) residents highlighted the role of host genetics in susceptibility for COVID-19 disease severity via polymorphism of key alleles that participate in the vitamin D metabolism pathway [30]. Potential contributory factors for vitamin D deficiency among Arabs includes darker skin pigmentation, which decreases dermal vitamin D synthesis and a preference for conservative dress in some cultures and religious societies, especially among women, which further decreases skin exposure to light and lower serum vitamin D level [31–33]. A recent study suggested an association between UVA or UVB exposure to COVID-19 disease severity independent of vitamin D [34].

The dietary patterns of Israeli Arabs, traditionally low in meat and fish dishes, also play an essential role in observed low vitamin D levels in this group [35, 36]. Additional potential causes for low vitamin D among Israeli Arabs may stem from delayed medical attention seeking in community settings, particularly for non-communicable diseases [37]. Potential medical disparities and late referrals to hospitals after symptoms onset may underlie the higher ratio of Israeli Arabs to non-Arabs Israelis among critical cases of COVID-19 in our cohort. Altogether, despite the significant propensity for vitamin D deficiency among Israeli Arabs, our data showed no effect of ethnicity on disease severity and mortality (Tables 1–3).

Preexisting medical conditions, healthcare accessibility, and socioeconomic factors may contribute to the disproportionate impact of COVID-19 on minority populations worldwide. A higher rate of COVID-19 positivity among the Black and Hispanic population in the US was attributed to low circulating vitamin D status but also to other, non-biological factors such as greater barriers to social distancing [38–40].

There are several important limitations of the study. First, vitamin D deficiency can be one indication of a wide range of chronic health conditions or behavioral factors that simultaneously increase COVID-19 disease severity and mortality risks. For example, COPD is a known risk factor for poorer COVID-19 outcomes with or without concurrent vitamin D deficiency [41]. Second, patients’ supplementation history was not obtained or analyzed as part of our research. The use of historical results from community health providers may be influenced by prior vitamin D deficiency correction therapy given due to low serum levels, the effect of which is difficult to fully deduce. However, our cohort’s strong correlation between prior vitamin D deficiency and COVID-19 disease outcome implies that most patients remain with low 25(OH)D values when contracting COVID-19 infection. Third, while our findings have identified an association between pre-infection vitamin D deficiency and COVID-19 severity, these results do not necessarily imply that vitamin D treatment will impact COVID-19 outcomes. Therefore, we should remain cautious about overestimating the potential benefit of vitamin D supplementation in improving outcomes of SARS-CoV-2 infection.

Existing literature suggests a potential protective effect of supplemental vitamin D in preventing and treating COVID-19 disease (reviewed in [42]). A published meta-analysis of 43 observational studies analyzing data obtained from 612,601 patients showed that vitamin D deficiency (defined as 25(OH)D of <20 ng/mL) increases the risk of acute COVID-19 infections compared with concentrations >30 ng/mL (odds ratio [OR], 1.26; 95% confidence interval [CI], 1.19 to 1.34; *p* < 0.01). One meta-analysis of three randomized controlled trials (RCTs) and two Quasi-experimental analyzing data obtained from 467 patients has raised doubt as to whether low vitamin D is associated with an increased risk of acquiring COVID-19 [43]. A more recent placebo-controlled, double-blind RCT tested the effect of calcifediol 25(OH)D3 treatment in 106 COVID-19 Iranian patients and found that an oral calcifediol treatment resulted in improved immune function with an increased blood lymphocyte percentage and reduced blood neutrophil-to-lymphocyte ratio compared to the placebo group [44]. An additional retrospective study found that prescription of calcifediol or vitamin D, 15–30 days before hospitalization with COVID-19 infections, was found to improved patient survival in a large retrospective, hospitalized, Andalusian cohort [45]. It should be emphasized that 25(OH)D represents only one piece of the complex puzzle that is the illness caused by COVID-19 in addition to underlying comorbidities, genetic predispositions, dietary habits, and geographic factors. Despite the numerous studies related to 25(OH)D and COVID-19, to date, more well-designed RCTs are required to address further the potential therapeutic applications of vitamin D for patients infected with SARS-CoV-2.

## Conclusion

From the early stages of the COVID-19 pandemic, establishing vitamin D deficiency as a risk factor was the aim of many investigators. It was subject to much debate in the general public and multiple medical journals [46]. Our study contributes to a continually evolving body of evidence that suggests a patient’s history of vitamin D deficiency is a predictive risk factor associated with poorer COVID-19 clinical disease course and mortality. The use of historical results obtained before the COVID-19 pandemic as part of a public health survey enabled us to suggest vitamin D deficiency contributes to the causal pathway of COVID-19 mortality risk and disease severity. Our study warrants further studies investigating if and when vitamin D supplementation among vitamin D deficient individuals in the community impacts the outcome of an eventual COVID-19 episode.

## Supporting information

S1 Dataset Demographic characteristics. (XLSX)
